# Fixed combination of oral NEPA (netupitant‐palonosetron) for the prevention of acute and delayed chemotherapy‐induced nausea and vomiting in patients receiving multiple cycles of chemotherapy: Efficacy data from 2 randomized, double‐blind phase III studies

**DOI:** 10.1002/cam4.2091

**Published:** 2019-04-09

**Authors:** Lee Schwartzberg, Meinolf Karthaus, Giorgia Rossi, Giada Rizzi, Maria E. Borroni, Hope S. Rugo, Karin Jordan, Vincent Hansen

**Affiliations:** ^1^ West Cancer Center Memphis Tennessee; ^2^ Staedt. Klinikum Neuperlach and Harlaching Munich Germany; ^3^ Helsinn Healthcare SA Lugano Switzerland; ^4^ University of California San Francisco Comprehensive Cancer Center San Francisco California; ^5^ Department of Medicine V, Hematology, Oncology and Rheumatology University of Heidelberg Germany; ^6^ Northern Utah Associates Ogden Utah

**Keywords:** CINV, delayed phase, efficacy, multiple cycles, NEPA, netupitant

## Abstract

**Aim:**

To assess the efficacy of oral NEPA (netupitant‐palonosetron 300/0.50 mg) over multiple chemotherapy cycles.

**Methods:**

Two randomized phase III studies evaluated a single dose of oral NEPA given on day 1 in chemotherapy‐naive patients receiving anthracycline‐cyclophosphamide (AC)–based (Study 1) or highly (HEC)/moderately (MEC) emetogenic chemotherapy (safety Study 2). Oral NEPA was compared with oral palonosetron 0.50 mg (Study 1) or oral aprepitant 125 mg day 1, 80 mg days 2‐3/palonosetron 0.50 mg (Study 2; no formal statistical comparisons). Oral dexamethasone was administered in all treatment groups. Complete response (CR; no emesis/no rescue medication), no emesis, and no significant nausea (NSN) rates during acute (0‐24 h) and delayed (>24‐120 h) phases of chemotherapy cycles 1‐4 in each study were evaluated.

**Results:**

In Study 1, 1450 patients received 5969 chemotherapy cycles; in Study 2, 412 patients received 1961 chemotherapy cycles. In each study, ≥75% of patients completed 4 or more cycles. In Study 1, oral NEPA was superior to palonosetron in preventing chemotherapy‐induced nausea and vomiting (CINV) in the acute and delayed phases of cycle 1, with higher rates of CR (all *P* < 0.05), no emesis (all *P* < 0.05), and NSN (delayed phase *P* < 0.05 cycles 1, 2, and 4) reported across 4 cycles. In Study 2, oral NEPA had numerically higher CR and NSN rates in the acute and delayed phases than aprepitant‐palonosetron in MEC/HEC patients.

**Conclusion:**

Oral NEPA was highly effective in preventing both acute and delayed CINV over multiple chemotherapy cycles of HEC, AC, and MEC regimens.

**Clinical trial registration numbers:**

Study 1, NCT01339260; Study 2, NCT01376297.

## 1 INTRODUCTION

Chemotherapy‐induced nausea and vomiting (CINV) is a debilitating complication and one of multiple adverse events frequently reported in patients receiving routine chemotherapy. If poorly controlled, CINV impairs quality of life^1^ and may compromise anticancer treatment adherence (reviewed in Hesketh^2^). Nausea and vomiting belong to a cluster of symptoms that if correctly managed, may lead to longer survival.^3^, ^4^ CINV is primarily mediated through neurotransmitters, such as serotonin, substance P, and dopamine,^5^ and can be categorized into acute (0‐24 h) and delayed phases (>24‐ 120 h).^2^ Acute CINV results mainly from serotonin's action on the 5‐hydroxytryptamine‐3 (5‐HT_3_) receptor, while delayed CINV is mainly mediated by substance P acting on the neurokinin‐1 (NK_1_) receptor.^6^

Delayed CINV occurs more frequently than acute CINV,^1^, ^7^ and is experienced by over 50% of patients receiving chemotherapy, despite antiemetic prophylaxis use.^1^, ^7^ It tends to be underreported by patients, and the incidence is underestimated by most oncology physicians and nurses.^7^, ^8^, ^9^

For effective antiemetic prophylaxis, control throughout the entire period of emetic risk in the first and subsequent chemotherapy cycles is necessary.^10^ If CINV is inadequately controlled in the first cycle, it may become more difficult to manage,^11^ with a 14% increased risk of CINV in subsequent cycles.^12^ Controlling CINV over multiple cycles with an NK_1_ receptor antagonist (RA) has been shown to reduce resource utilization, particularly by preventing delayed CINV.^13^, ^14^ Prevention of CINV from the first cycle therefore remains the main goal for successful CINV control.

Current antiemetic guidelines of the National Comprehensive Cancer Network (NCCN)^15^ and the Multinational Association of Supportive Care in Cancer (MASCC)/European Society for Medical Oncology (ESMO)^16^ recommend the triplet combination of an NK_1_ RA, a 5‐HT_3_ RA, and dexamethasone (DEX) to prevent CINV in patients receiving highly emetogenic chemotherapy (HEC).^15^, ^16^, ^17^ The American Society of Clinical Oncology (ASCO) and NCCN endorse the addition of olanzapine to this triplet in patients receiving HEC and before the start of chemotherapy, with additional prophylaxis (DEX and olanzapine) on days 2‐4 of chemotherapy; NK_1_ RA aprepitant (APR) is part of the prophylaxis on days 2‐3 if given on day 1.^15^, ^17^ For patients receiving moderately emetogenic chemotherapy (MEC), a 5‐HT_3_ RA in combination with DEX on day 1 is generally advised,^15^, ^16^, ^17^ with the addition of an NK_1_ RA for certain patients with additional risk factors or previous treatment failure when receiving a steroid plus 5‐HT_3_ RA alone^15^; additional prophylaxis may be offered on days 2 and 3 of chemotherapy if necessary.^15^, ^17^ MASCC/ESMO first introduced a new recommendation for adding an NK_1_ RA to the 5‐HT_3_ RA plus DEX regimen for patients receiving carboplatin, regardless of dose.^16^ The NCCN and ASCO guidelines now also make the same recommendation for carboplatin area under the curve (AUC) ≥4 mg mL^−1^ minied carboplatin.^15^, ^17^ Only the NCCN guidelines have reclassified carboplatin AUC ≥4 mg mL^−1^ min from a MEC to a HEC agent.^15^

Oral NEPA is the first and only antiemetic combination agent; it is composed of netupitant (300 mg), a highly selective NK_1_ RA, and the pharmacologically^18^ and clinically^19^ distinct 5‐HT_3_ RA palonosetron (PALO, 0.50 mg). NEPA thereby antagonizes 2 key neurotransmitters involved in the pathophysiology of CINV, and provides acute and delayed CINV control with a single dose. Real‐world evidence suggests complicated antiemetic schedules are often not followed by patients, leading to mistakes/missed doses of prophylactic agents prescribed to be taken over multiple days.^5^ The convenient administration schedule of oral NEPA may therefore enable improved adherence to the antiemetic regimen and guidelines. Oral NEPA has been shown to be superior to oral PALO in preventing CINV during the acute, delayed, and overall phases following the first cycle of cisplatin‐based^20^ or anthracycline‐cyclophosphamide (AC)‐based chemotherapy.^21^ Oral NEPA is well tolerated, with a safety profile consistent with the NK_1_ RA and 5‐HT_3_ RA classes.^20^, ^21^ An intravenous (IV) formulation of the NEPA fixed combination has been developed to offer clinicians and patients further convenience, and IV NEPA plus DEX was recently approved by the US Food and Drug Administration for the prevention of CINV in patients receiving HEC, with a limitation of use in AC‐based chemotherapy.^22^ A phase IIIb study evaluating the safety of IV NEPA in patients receiving AC‐based chemotherapy is ongoing.

Two phase III studies, evaluating the efficacy and safety of oral NEPA over multiple cycles of chemotherapy, form the basis of this report.^21^, ^23^, ^24^ In both studies, previously published data demonstrated that oral NEPA maintained antiemetic control during the 5‐day period following chemotherapy (overall phase) over at least 4 cycles of chemotherapy.^23^, ^24^ Oral NEPA also showed superior complete response (CR) rates compared with oral PALO during the overall phase in cycle 1, and the difference was statistically significant over repeated cycles.^23^ At the time both trials were conducted, MEC included AC‐based regimens in patients with breast cancer (referred to herein as AC MEC). However, AC‐based chemotherapy has since been reclassified as HEC.^15^, ^16^, ^17^ For consistency with the original publications of each trial, patients are referred to as receiving AC MEC in Study 1^21^ and HEC or non‐AC MEC in Study 2 (breast cancer patients scheduled to receive AC‐based chemotherapy in Study 2 were not eligible).^24^ This report focuses on the efficacy of oral NEPA during the acute and delayed phases over 4 cycles of chemotherapy in these studies.

## 2 METHODS

### 2.1 Studies

Two international, randomized, double‐blind phase III trials, Study 1 (NCT01339260)^21^ and Study 2 (NCT01376297),^24^ were analyzed. Both evaluated the efficacy of oral NEPA in patients with solid tumors, including patients diagnosed with any malignant tumor in Study 2. Detailed study designs, methods, and eligibility criteria have been reported previously and are summarized in Figure 1.^21^, ^24^ Oral DEX was open‐label and the dosing schedule was based on the emetogenicity of the chemotherapy according to the antiemetic guidelines valid at the time the studies were performed.^25^ Both study protocols were approved by the relevant ethical review committees, all patients provided written informed consent, and all investigators and site personnel followed International Conference on Harmonization E6 Good Clinical Practice guidelines, Declaration of Helsinki (2008) ethical principles, and local laws and regulations.

**Figure 1:** Schemas of 2 international, randomized, double‐blind phase III trials: Study 1 (NCT01339260)^21^ and Study 2 (NCT01376297).^24^ ^a^3:1 randomization NEPA: APR + PALO; the protocol also specified that 75% of patients would receive MEC and 25% HEC. AC, anthracycline‐ cyclophosphamide; APR, aprepitant; DEX, dexamethasone; HEC, highly emetogenic chemotherapy; MEC, moderately emetogenic chemotherapy; NEPA, netupitant‐palonosetron; NETU, netupitant; PALO, palonosetron

### 2.2 Assessments

CR (defined as no emesis and no rescue medication) and no significant nausea (NSN; defined as a score of <25 mm on a visual analog scale of 100 mm) were assessed during the acute and delayed phases after chemotherapy initiation, for the first 4 cycles; “no emesis” was also collected in Study 1.

### 2.3 Statistical considerations

Efficacy data were not pooled across the 2 studies because of different study objectives, designs, chemotherapy regimens, and populations. All efficacy analyses were undertaken on the full analysis set (defined as all randomized patients who received chemotherapy and study drug). In Study 1, CR, no emesis, and NSN rates for the oral NEPA and oral PALO arms were compared using a 2‐sided Cochran‐Mantel‐Haenszel test stratified by age class (<55 years, ≥55 years) and region (US, Latin America, Europe, Commonwealth of Independent States, and Asia) for all 4 cycles; this test was the same used at cycle 1 for the primary and key secondary efficacy analyses as per prespecified study plan. For cycles 2‐4, a formal statistical comparison was not prespecified; no method to adjust for multiplicity was applied. No formal comparisons of efficacy were made between the oral NEPA and oral APR‐PALO arms in Study 2, as its primary endpoint was safety. CR and NSN rates are also reported separately for the subsets of NEPA patients receiving either MEC or HEC; APR‐PALO data are not included for these chemotherapy subsets since the small sample size (considering the 3:1 randomization ratio) hindered interpretation, especially for repeated cycles. As most patients completed their planned therapy after 4 treatment cycles, efficacy data are presented over only cycles 1‐4 (safety data have been previously published^21^).

## 3 RESULTS

### 3.1 Analyzed patient population

In total, 1455 patients were randomized in Study 1: 726 to oral NEPA and 729 to oral PALO (Table 1). Of these, 1450 patients (99.7%) were treated for a total of 5969 chemotherapy cycles; 1438 patients (98.8%) completed cycle 1, and 1286 patients (88.4%) entered the multiple‐cycle extension 23; 1107 patients (76.1%) completed 4 or more cycles. Most patients completed their planned chemotherapy after 4 treatment cycles; 35.7% of patients received a fifth cycle, and 26.7% received a sixth cycle (data not shown).

**Table 1:** Summary of patient disposition from Study 1 and Study 2—all randomized patients

	Study 1^a^			Study 2^b^		
	NEPA (N = 726) (C = 2983)	PALO (N = 729) (C = 2986)	Overall (N = 1455) (C = 5969)	NEPA (N = 309) (C = 1446)	APR‐PALO (N = 104) (C = 515)	Overall (N = 413) (C = 1961)
Treated, n (%)	724 (99.7)	726 (99.6)	1450 (99.7)	309 (100.0)	103 (99.0)	412 (99.8)
Completed cycle 1, n (%)	719 (99.0)	719 (98.6)	1438 (98.8)	303 (98.1)	102 (98.1)	405 (98.1)
Completed cycle 2, n (%)	630 (86.8)	645 (88.5)	1275 (87.6)	278 (90.0)	94 (90.4)	372 (90.1)
Completed cycle 3, n (%)	596 (82.1)	603 (82.7)	1199 (82.4)	255 (82.5)	88 (84.6)	343 (83.1)
Completed cycle 4, n (%)	548 (75.5)	559 (76.7)	1107 (76.1)	230 (74.4)	81 (77.9)	311 (75.3)

C = Total number of cycles started for all treated patients.

APR, aprepitant; NEPA, netupitant‐palonosetron; PALO, palonosetron.

a Data corresponding to cycles 5‐8 not shown.

b Data corresponding to cycles 5‐14 not shown.

In Study 2, 413 patients were randomized: 309 to oral NEPA and 104 to oral APR‐PALO (Table 1). Of these, 412 patients (99.8%) were treated for a total of 1961 chemotherapy cycles; 405 patients (98.1%) completed cycle 1, 311 patients (75.3%) completed 4 or more cycles; 51.6% of patients received a fifth cycle, and 40.0% received a sixth cycle (data not shown).

Baseline and disease characteristics from both studies are reported in Table 2. These characteristics remained consistent across cycles, and were similar between treatment arms. In Study 1, the median age was 54 years, 98.1% of patients were female, and 97.4% had breast cancer. In Study 2, the median age was 58 years, 50% of patients were female, and the most prevalent cancer was lung/respiratory cancer (37.4%). Per protocol, most patients (75.7%) received MEC (Table 3).

**Table 2:** Baseline and disease characteristics of patients from Study 1 and Study 2—safety population (cycle 1)

	Study 1			Study 2		
	NEPA (N = 725)	PALO (N = 725)	Overall (N = 1450)	NEPA (N = 308)	APR‐PALO (N = 104)	Overall (N = 412)
Gender, %						
Male	1.9	1.9	1.9	49.7	51.0	50.0
Female	98.1	98.1	98.1	50.3	49.0	50.0
Median age, years	54.0	54.0	54.0	57.0	58.5	58.0
Cancer type, %						
Breast	97.7	97.2	97.4	12.7	8.7	11.7
Lung/respiratory	—	—	—	39.6	30.8	37.4
Ovarian	—	—	—	10.7	17.3	12.4
Head and neck	—	—	—	6.5	10.6	7.5
Colorectal	—	—	—	16.2	22.1	17.7
Gastric	—	—	—	2.3	1.0	1.9
Bladder	—	—	—	1.3	2.9	1.7
Other^a^	2.3	2.8	2.6	16.7	6.7	9.7
Extent of cancer at entry, %						
Primary	81.8	82.9	82.3	43.8	51.9	45.9
Metastatic	16.3	15.6	15.9	51.9	43.3	49.8
Local recurrence	1.9	1.5	1.7	4.2	4.8	4.4
Site of metastasis, %						
Lymph nodes	10.8	11.7	11.2	33.1	21.2	30.1
Other	5.5	3.2	4.3	15.6	19.2	16.5
Liver	2.9	2.1	2.5	12.0	12.5	12.1
Bone	3.7	3.6	3.7	5.8	4.8	5.6
Brain	0.3	0	0.1	1.6	2.9	1.9
ECOG performance status, %						
1	69.5	69.2	69.4	47.4	48.1	47.6
2	29.7	30.6	30.1	51.0	50.0	50.7
3	0.8	0.1	0.5	1.6	1.9	1.7

APR, aprepitant; ECOG, Eastern Cooperative Oncology Group; NEPA, netupitant‐palonosetron; PALO, palonosetron.

a The category “other” included any other type of cancer not listed in the prespecified categories, including, but not limited to, those of the uterus, larynx, and endometrium.

**Table 3:** Chemotherapy received in patients from Study 1 and Study 2—safety population (cycle 1)

Study 1 chemotherapy^a^, %	NEPA (N = 725)	PALO (N = 725)	Overall (N = 1450)
AC^b^			
Doxorubicin	68.0	63.6	65.8
Cyclophosphamide	99.9	99.9	99.9
Epirubicin	32.0	36.3	34.2

Study 2 chemotherapy^a^, %	NEPA (N = 308)	APR‐PALO (N = 104)	Overall (N = 412)
MEC^c^	75.7	75.7	75.7
Carboplatin	60.3	61.5	60.6
Oxaliplatin	20.1	24.4	21.2
Doxorubicin^d^	11.1	6.4	9.9
Cyclophosphamide^d^	3.4	2.6	3.2
Irinotecan	3.0	3.8	3.2
Epirubicin^d^	1.7	1.3	1.6
Daunorubicin	0.4	0	0.3
HEC^c^	24.3	24.3	24.3
Cisplatin	96.0	92.0	95.0
Dacarbazine	4.0	4.0	4.0
Carmustine	0	4.0	1.0

AC, anthracycline‐cyclophosphamide; APR, aprepitant; HEC, highly emetogenic chemotherapy; MEC, moderately emetogenic chemotherapy; NEPA, netupitant‐palonosetron, PALO: palonosetron.

a Percentages are based on efficacy (full analysis) population, while all others are based on safety population (cycle 1).

b Breast cancer patients scheduled to receive AC‐based chemotherapy in Study 2 were not eligible.

c Cycle 1 chemotherapy.

d Cyclophosphamide and doxorubicin or epirubicin were administered together as “AC” in Study 1.

### 3.2 Efficacy

#### 3.2.1 Study 1

Oral NEPA was superior to oral PALO in preventing CINV in the acute and delayed phases in cycle 1 (Table 3, Figure 2A), with high rates of control maintained in subsequent cycles. In the oral NEPA group, CR rates ranged from 88.4% to 91.6%, and 76.9% to 85.5% for the acute and delayed phases, respectively, across 4 cycles. These rates were higher and differences were statistically significant compared with the PALO group (between‐group comparisons for individual cycles, all *P* < 0.05 not adjusted for multiplicity). Likewise, higher rates of NSN and no emesis were observed for oral NEPA versus oral PALO (Table 4). In the oral NEPA group, the rates of no emesis across 4 cycles ranged from 90.9% to 93.1%, and 81.8% to 89.5% for the acute and delayed phases, respectively, and differences were statistically significant compared with the PALO‐treatment group (between‐group comparisons for individual cycles, all *P* < 0.05 not adjusted for multiplicity). In the oral NEPA group, the rates of NSN across 4 cycles ranged from 87.3% to 91.3%, and 76.9% to 81.7% for the acute and delayed phases, respectively; differences were statistically significant in the delayed‐phase NSN rates compared with the PALO group (between‐group comparisons for individual cycles, *P* < 0.05 for cycles 1, 2, and 4 not adjusted for multiplicity).

**Figure 2:** CR (no emesis, no rescue medication) rates in the delayed phase (>24‐120 h) of cycles 1‐4 in: A) Study 1 (patients receiving AC‐based chemotherapy), and B) Study 2 (patients receiving HEC or MEC^a^). Full analysis set. ^a^Breast cancer patients were not allowed AC‐based regimens. AC, anthracycline‐cyclophosphamide; APR, aprepitant; CR, complete response; HEC, highly emetogenic chemotherapy; MEC, moderately emetogenic chemotherapy; NEPA, netupitant‐palonosetron; PALO, palonosetron

**Table 4:** CR, no emesis, and NSN rates in the acute (0‐24 h) and delayed (>24‐120 h) phase of cycles 1‐4—full analysis set

Study 1	Cycle (N = NEPA/PALO)		Cycle 1 (N = 724/725)	Cycle 2 (N = 635/651)	Cycle 3 (N = 598/606)	Cycle 4 (N = 551/560)
CR	Acute	NEPA, %	88.4	89.9	91.6	91.5
		PALO, %	85.0	83.7	83.8	86.8
		*P* value^a^	0.047	0.001	<0.001	0.011
	Delayed	NEPA, %	76.9	81.7	85.1	85.5
		PALO, %	69.5	68.8	74.4	77.3
		*P* value^a^	0.001	<0.001	<0.001	<0.001
	Overall	NEPA, %	74.3	80.3	83.8	83.8
		PALO, %	66.6	66.7	70.3	74.6
		*P* value^a^	0.001	<0.001	<0.001	<0.001
No emesis	Acute	NEPA, %	90.9	92.6	93.0	93.1
		PALO, %	87.3	86.8	87.5	88.4
		*P* value^a^	0.025	<0.001	0.002	0.006
	Delayed	NEPA, %	81.8	86.3	89.5	88.8
		PALO, %	75.6	76.5	81.0	82.3
		*P* value^a^	0.004	<0.001	<0.001	0.002
	Overall	NEPA, %	79.8	85.5	88.3	87.3
		PALO, %	72.1	73.7	77.2	79.5
		*P* value^a^	<0.001	<0.001	<0.001	<0.001
NSN^b^	Acute	NEPA, %	87.3	88.8	89.1	91.3
		PALO, %	87.9	87.3	87.1	88.9
		*P* value	0.747	0.431	0.297	0.181
	Delayed	NEPA, %	76.9	79.5	79.8	81.7
		PALO, %	71.3	74.0	75.4	76.4
		*P* value^a^	0.014	0.017	0.062	0.025
	Overall	NEPA, %	74.6	77.3	78.4	80.2
		PALO, %	69.1	71.6	73.3	75.2
		*P* value^a^	0.020	0.016	0.033	0.035

Study 2	Cycle (N = NEPA/APR + PALO)		Cycle 1 (N = 309/103)	Cycle 2 (N = 280/96)	Cycle 3 (N = 259/90)	Cycle 4 (N = 233/81)
CR	Acute	NEPA, %	92.9	96.4	96.1	96.6
		APR + PALO, %	94.2	91.7	95.6	96.3
	Delayed	NEPA, %	83.2	86.8	91.5	91.0
		APR + PALO, %	77.7	82.3	87.8	87.7
	Overall	NEPA, %	80.6	86.1	90.7	90.1
		APR + PALO, %	75.7	81.3	86.7	87.7
NSN^b^	Acute	NEPA, %	90.6	95.4	96.1	97.0
		APR + PALO, %	93.2	92.7	93.3	95.1
	Delayed	NEPA, %	85.1	87.5	90.0	91.8
		APR + PALO, %	81.6	86.5	84.4	86.4
	Overall	NEPA, %	84.1	86.8	89.6	91.8
		APR + PALO, %	80.6	86.5	83.3	86.4

APR, aprepitant; CR, complete response; NEPA, netupitant‐palonosetron; NSN, no significant nausea; PALO, palonosetron; VAS, visual analog scale.

a Test prespecified and adjusted for multiplicity for CR at cycle 1 only; post‐hoc for cycles 2‐4 (not adjusted for multiplicity).

b Defined as maximum daily nausea score <25 mm on 100‐mm VAS.

#### 3.2.2 Study 2

In Study 2, the CR rates were high across cycles 1‐4 for both treatment groups. In patients treated with oral NEPA, CR rates ranged from 92.9% to 96.6%, and 83.2% to 91.5% for the acute and delayed phases, respectively. These rates were similar but numerically higher compared with oral APR‐PALO, except for acute CR and acute NSN in cycle 1 (Table 4, Figure 2B). Similar results were seen in the subsets of NEPA patients receiving MEC (n = 235 at cycle 1). Across cycles 1‐4, CR rates of 93.2%, 97.2%, 96.4%, and 97.2% were observed in the acute phase, and 81.7%, 88.7%, 90.8%, and 91.7% in the delayed phase. For APR‐PALO patients receiving MEC (n = 77 at cycle 1), CR rates of 93.5%, 94.6%, 97.3%, and 97.0% were observed across cycles 1‐4 in the acute phase, and 84.4%, 85.1%, 87.8%, and 88.1% in the delayed phase (data not shown). For the subset of NEPA patients receiving HEC (n = 74 at cycle 1), CR rates of 91.9%, 94.1%, 95.2%, and 94.2% were reported across cycles 1‐4 in the acute phase, and 87.8%, 80.9%, 93.7%, and 88.5% in the delayed phase. For APR‐PALO patients receiving HEC (n = 26 at cycle 1), CR rates of 96.2%, 81.8%, 87.5%, and 92.9% were reported across cycles 1‐4 in the acute phase, and 57.7%, 72.7%, 87.5%, and 85.7% in the delayed phase (data not shown).

NSN rates were also high in both treatment groups, with numerically higher rates for NEPA compared with APR‐PALO. Across cycles 1‐4, NEPA‐treated patients had NSN rates ranging from 90.6% to 97.0%, and 85.1% to 91.8% in the acute and delayed phases, respectively (Table 4).

## 4 DISCUSSION

This report presents the efficacy results of 2 pivotal trials evaluating the safety and efficacy of oral NEPA in the acute and delayed phases over multiple chemotherapy cycles in patients with solid tumors (in Study 2, patients with any malignant tumor were eligible). In Study 1, superiority of NEPA to PALO in preventing CINV in the acute, delayed, and overall phases during cycle 1 of AC‐based chemotherapy was clearly demonstrated,^21^ with overall CR sustained across multiple cycles^23^ (overall CR for oral NEPA was 74.3%–83.8% across 4 cycles; overall no emesis and NSN rates for oral NEPA were 79.8%–88.3% and 74.6%–80.2%, respectively, all across 4 cycles [Table 3]). The current analysis now reports higher response rates with NEPA, compared with PALO, for all 3 efficacy measures (CR, NSN, and no emesis) during the acute and delayed phases across all 4 chemotherapy cycles (*P* < 0.05 not adjusted for multiplicity). In the previously reported results of Study 2, the safety and efficacy with NEPA were maintained, and NEPA resulted in numerically higher overall CR rates than APR‐PALO in cycle 1 and subsequent cycles^24^ (overall CR for oral NEPA was 80.6%–90.7% across 4 cycles; overall NSN for oral NEPA was 84.1%–91.8% across 4 cycles [Table 3]). This current analysis also found CR and NSN rates were numerically higher for NEPA in the acute and delayed phases for both the overall population and the MEC and HEC subgroups.

Collectively, these data show the efficacy of oral NEPA in preventing CINV, particularly in the delayed phase in cycle 1; this was maintained over multiple cycles. NK_1_ RA regimens have historically been studied primarily in cisplatin‐based HEC and AC settings, so these data expand the known efficacy of NEPA, ergo NK_1_ RA regimens, to MEC regimens as well. These findings are thus relevant to a broad range of chemotherapeutic settings, which is important considering the recent reclassification in the guidelines of carboplatin AUC ≥ 4^15^ and AC combination regimens to HEC.^15^, ^16^, ^17^

The high NSN rates are notable given the unmet clinical need for CINV prevention in the delayed setting, particularly for nausea control.^26^ Evidence from phase III studies of APR showed “no nausea” rates between 44% and 71%, and NSN rates between 57% and 78% in the delayed phase.^27^, ^28^, ^29^, ^30^, ^31^ A study of the NK_1_ RA rolapitant added to a granisetron‐DEX regimen reported no statistically significant improvement to nausea control in patients receiving AC and non‐AC HEC.^32^ Another pooled analysis of 2 studies in patients receiving cisplatin‐based HEC reported statistically higher rates of NSN and “no nausea” in patients receiving rolapitant‐granisetron‐DEX, compared with those receiving granisetron‐DEX alone. However, when analyzed separately, 1 of the 2 trials showed no statistically significant difference in NSN rates.^33^ Another study reported statistically significantly higher NSN but not “no nausea” rates in patients receiving rolapitant‐ondansetron‐DEX compared with ondansetron‐DEX with cisplatin‐based HEC.^34^

Each of the 2 studies in this analysis reported more than 3‐quarters of patients evaluable at the end of cycle 4. This is in contrast to other studies investigating antiemetic usage across multiple cycles. A recent post‐hoc analysis of pooled efficacy data from 4 trials of rolapitant presenting data from 2637 patients undergoing up to 6 cycles of chemotherapy reported that only ~50% completed cycle 4.^35^ Other multiple‐cycle trials of antiemetics also reported high dropout rates, which has hampered the interpretation of results in these studies.^36^, ^37^, ^38^, ^39^, ^40^ Despite NEPA's sustained efficacy over multiple cycles reported in the present analysis, there are limitations to our methodology. The 2 studies were sufficiently heterogeneous, preventing pooled analysis, and the main focus of Study 2 was on safety, hence not designed to formally compare the efficacy of oral NEPA with an APR triplet (the APR‐PALO arm was included only as a safety reference). Furthermore, the increased percentage of patients in both studies with CR and NSN in subsequent cycles may reflect a selection bias in which responders, but not nonresponders, preferentially continued to receive further cycles. In the subset of patients treated with MEC, 60% of patients received carboplatin. It is noteworthy that carboplatin was considered as MEC by all guidelines at the time the study was conducted; however, all guidelines currently recommend antiemetics consistent with those administered for HEC in patients receiving carboplatin AUC ≥ 4 mg mL^−1^ min.

In conclusion, oral NEPA, the first antiemetic combination agent targeting 2 critical emetic pathways, demonstrated superiority over PALO in terms of CR in all 3 phases of cycle 1 (Study 1); also, NEPA resulted in high CR and NSN rates during the acute and delayed phases, as well as in the overall phase across the 4 cycles (Studies 1 and 2), regardless of whether patients were receiving an AC MEC, non‐AC MEC, or HEC regimen. Preservation of the antiemetic effect of oral NEPA over multiple cycles suggests the utility of this agent in providing sustained CINV control beyond the first cycle. The convenient fixed single‐dose, once‐per‐cycle administration of oral NEPA may improve adherence to antiemetic guidelines and increase treatment compliance, hence improve CINV prevention; this will need to be verified in prospective studies.

## CONFLICT OF INTEREST

The authors have the following conflicts of interest to disclose: LS: consultant for Helsinn Healthcare, Tesaro, Merck, and Heron. MK: consultant for Helsinn Healthcare, MSD, and Tesaro. GRo, GRi, and MEB: employees of Helsinn Healthcare. HSR: research funding from UCSF and Eisai. KJ: consultant or received honoraria from Helsinn Healthcare, Tesaro, and Merck/MSD. VH: none declared.
